This article has been retracted.

# Critical role of CCDC6 in the neoplastic growth of testicular germ cell tumors

**DOI:** 10.1186/1471-2407-13-433

**Published:** 2013-09-24

**Authors:** Stefania Staibano, Gennaro Ilardi, Vincenza Leone, Chiara Luise, Francesco Merolla, Francesco Esposito, Francesco Morra, Maria Siano, Renato Franco, Alfredo Fusco, Paolo Chieffi, Angela Celetti

**Affiliations:** 1 Istituto di Endocrinologia ed Oncologia Sperimentale, CNRz, via S Pansini, 5, Naples 80131, Italy; 2 Dipartimento di Medicina Molecolare e Biotecnologie Mediche, Università Federico II, Naples, Italy; 3 Dipartimento di Scienze Biomediche Avanzate, Università Federico II, Naples, Italy; 4 ISNT G. Pascale, Naples, Italy; 5 Dipartimento di Psicologia, Seconda Università di Napoli, Caserta 81100, Italy

**Keywords:** CCDC6, Testicular germ cells tumours, TMA, DNA damage response, T-CAM2, GC-1, ROS, Oxidative DNA damage

## Abstract

**Background:**

DNA damage response has been clearly described as an anti-cancer barrier in early human tumorigenesis. Moreover, interestingly, testicular germ cell tumors (TGCTs) have been reported to lack the DNA Damage Response (DDR) pathway activation.

CCDC6 is a pro-apoptotic phosphoprotein substrate of the kinase ataxia telangectasia mutated (ATM) able to sustain DNA damage checkpoint in response to genotoxic stress and is commonly rearranged in malignancies upon fusion with different partners.

In our study we sought to determine whether CCDC6 could have a role in the patho-genesis of testicular germ cell tumors.

**Methods:**

To achieve this aim, analysis for CCDC6 expression has been evaluated on serial sections of the mouse testis by immunohistochemistry and on separate populations of murine testicular cells by western blot. Next, the resistance to DNA damage-induced apoptosis and the production of reactive oxygen species has been investigated in GC1 cells, derived from immortalized type B murine germ cells, following CCDC6 silencing. Finally, the CCDC6 expression in normal human testicular cells, in Intratubular Germ Cell Neoplasia Unclassified (IGCNU), in a large series of male germ cell tumours and in the unique human seminoma TCam2 cell line has been evaluated by immunohistochemistry and by Western Blot analyses.

**Results:**

The analysis of the CCDC6 expression revealed its presence in Sertoli cells and in spermatogonial cells. CCDC6 loss was the most consistent feature among the primary tumours and TCam2 cells. Interestingly, following treatment with low doses of H_2_O_2_, the silencing of CCDC6 in GC1 cells caused a decrease in the oxidized form of cytochrome c and low detection of Bad, PARP-1 and Caspase 3 proteins. Moreover, in the silenced cells, upon oxidative damage, the cell viability was protected, the γH2AX activation was impaired and the Reactive Oxygen Species (ROS) release was decreased.

**Conclusions:**

Therefore, our results suggest that the loss of CCDC6 could aid the spermatogonial cells to be part of a pro-survival pathway that helps to evade the toxic effects of endogenous oxidants and contributes to testicular neoplastic growth.

## Background

Testicular germ cell tumours (TGCTs), the most common malignancy in males aged 15–34 years, represent a major cause of death attributable to cancer in this age group [1,2]. TGCTs can be subdivided into seminoma and non-seminoma germ cell tumours (NSGCTs), including embryonal cell carcinoma, choriocarcinoma, yolk sac tumour and teratoma. Neoplasms containing more than one tumour cell component, eg seminoma and embryonal cell carcinoma, are referred to as mixed germ cell tumours. Seminomas and NSGCTs present distinctive clinical features with significant differences in prognosis and therapeutic approach [3]. Nevertheless, the molecular alterations and biomarkers of TGCTs still remain poorly defined [4]. Recently, it has been suggested that resistance to oxidative DNA damage is commonly associated to testicular germ cell transformation [5].

The maintenance of the genome integrity and the protection against the harmful mutagenic effects of DNA damage rely on the DNA damage response (DDR) machinery postulated to serve as an inducible barrier against tumorigenic transformation and/or progression for human cancers [6,7]. Notably, testicular germ cell tumours have been shown, so far, to represent an exception among human malignancies tested for constitutive DDR activation in that this phenomenon occurs only rarely [8].

In previous works we have documented the CCDC6 gene product as a pro-apoptotic protein substrate of ATM, able to sustain DNA damage checkpoints in response to DNA damage [8-10]. CCDC6 was originally identified upon rearrangement with RET in thyroid and lung tumours [11,12], and with genes other than RET in solid and not solid tumours [13-16]. In most cancers harbouring CCDC6 gene rearrangements, the product of the normal allele is supposed to be functionally impaired or absent. Fusions including CCDC6 or other genes have not been reported in TGCTs, so far (http://www.sanger.ac.uk/genetics/CGP/cosmic). Recently, the finding that CCDC6 helps to protect genome integrity by modulating PP4C activity directed towards pS139_H2AX dephosphorylation following DNA damage [11], makes CCDC6 an attractive candidate that could help pre-cancerous cells overcome a DNA damage response-dependent barrier against tumour progression. Therefore, we hypothesize that, when CCDC6 is deleted or silenced, the loss of checkpoints and of repair accuracy [17] might favour genome instability and may represent an early independent event of a multistep carcinogenetic process in primary tumours.

The tissue distribution and cell type-related expression patterns of CCDC6 in normal tissue remain largely unknown; on the other hand there are as yet no reports of analyses of CCDC6 in either human or animal tumours.

By the analysis of the Gene Expression Atlas (Array ExpressAtlas), a meta-analysis-based database of the ArrayExpress Archive, we noticed that CCDC6 was predicted as downregulated in germ cell tumours. Here, we intend to gain more insights into the CCDC6 tissue biology and its relation to testicular cancer in order to unravel a role for CCDC6 as a new DDR component that participates in genome stability maintenance and whose malfunction may contribute to the pathogenesis of germ cell tumours.

## Methods

### Cell lines and antibodies

The GC-1 cell line was cultured in Dulbecco’s modifiedEagle’s medium (D-MEM) supplemented with 10% fetal bovine serum (FBS; Gibco BRL, Italy) and grown in a 37°C humidified atmosphere of 5% CO2 [18]. TCAM-2 cells were grown at 37°C in a 5% CO2 atmosphere in RPMI 1640 (Lonza) supplemented with 10% FBS [19]. Anti pS139_H2AX antibody was from Millipore; Anti-H2AX, anti-pT68Chk2 and anti-Chk2 antibodies were from Cell Signaling Technology, Inc; anti MDC1 and anti CCDC6 were from Abcam; Anti-Cytochrome c (Biovision Inc, USA); anti COX IV (Cell Signaling Technology, Inc); Anti-Caspase 3 (H-277) Sc 7148, anti-Bcl 2 (N19) Sc 492, anti-PARP (H250) Sc 7150, anti-Bad (C20) Sc493 and secondary antibodies were from Santa Cruz Biotechnology, Inc; Anti α-tubulin was from Sigma -Aldrich Co. LLC.

### Plasmids and transfections

Mission shRNA (pLKO.1 puro) were from Sigma-Aldrich, Co. LLC.

For transient transfection assays the GC1 cells were transfected with the plasmid pool (shCCDC6, NM_001111121.1) or a pool of non- targeting vectors (sh control) by the Nucleofector transfection system. pCDNA4TO-CCDC6T434A mutant has been described elsewhere [10]. The Fugene reagent (Roche Ltd, Basel, Switzerland) was used to transfect GC1 cells accordingly to the manufacturer’s instructions.

### MTT cell proliferation assay

GC-1 cells were transfected with mission shCCDC6 or a control non-targeting scrambled sh, after 48h were treated with H_2_O_2_ at different doses (range of 1, 2, 5 and 10 μM) for 1h, as indicated. After washing out the hydrogen peroxide we have left the cells an additional hour before processing them. 20 ml of Promega’s CellTiter 96 AQueous One Solution (Promega) were then dispensed into each well and absorbance at 595 nm was measured to evaluate cell viability. Data reported are the average +/− s.d. of three independent experiments performed in sextuplicate. Anti-proliferative assays with a wide range of H_2_O_2_ doses (1, 2, 5, 10 and 50 μM) and at different times (30 min and 1 hour) in GC1 cells, transiently silenced, (shCCDC6 and shCtrl), are shown in the Additional file 1: Figure S1. Data reported are the average +/− s.d. of three independent experiments performed in sextuplicate.

### Apoptosis assays

GC-1 cells were transfected with mission shCCDC6 or a control non-targeting scrambled sh, after 48 h this cells were treated with H_2_O_2_ at 10 μM for 1 h and apoptosis was quantified by measuring Caspase 3/7 activation using the Caspase-Glo 3/7 assay (Promega) according to the manufacturer’s instructions.

### Cytochrome c releasing apoptosis assay Kit

GC-1 cells were transfected with mission shCCDC6 or a control non-targeting scrambled sh, after 48 h of transfection the apoptosis was induced by treatment of cells with H_2_O_2_ at 10 μM. After 1 h of H_2_O_2_ treatment, the cytochrome c release was quantified using the Cytochrome c Releasing Apoptosis Assay Kit (BioVision Inc, USA) according to the manufacturer’s instructions.

### Preparation of testicular cells

Germ cells were prepared from testes of adult CD1 mice (Charles River Italia). Testes were freed from the albuginea membrane and digested for 15 min in 0.25% (w/v) collagenase (type IX, Sigma) at room temperature under constant shaking. They were then washed twice in minimum essential medium (Life Technologies, Inc.), seminiferous tubules were cut into pieces with a sterile blade and further digested in minimum essential medium containing 1 mg/ml trypsin for 30 min at 30°C. Digestion was stopped by adding 10% fetal calf serum and the germ cells released were collected after sedimentation (10 min at room temperature) of tissue debris. Germ cells were centrifuged for 13 min at 1500 r.p.m. at 48°C and the pellet resuspended in 20 ml of elutriation medium (120.1 mM NaCl, 4.8 mM KCl, 25.2 mM NaHCO3, 1.2 mM MgS4 (7H2O), 1.3 mM CaCl2, 1.1 mM glucose, 1X essential amino acid (Life Technologies, Inc.), penicillin, streptomycin, 0.5% bovine serum albumin). Pachytene spermatocyte and spermatid germ cells were obtained by elutriation of the unfractionated single cell suspension. Homogeneity of cell populations ranged between 80 and 85% (pachytene spermatocytes) and 95% (spermatids), was routinely monitored morphologically. Spermatogonia were obtained from prepuberal mice as previously described [20]. Mature spermatozoa were obtained from the cauda of the epididymis of mature mice as described previously [21].

### TMA building

According to ethical guidelines, Tissue Micro-Array (TMA) was built using the most representative areas from each single case. All tumours and controls were reviewed by two experienced pathologists. Discrepancies between two pathologists from the same case were resolved in a joint analysis of the cases. Tissue cylinders with a diameter of 0.3 mm were punched from morphologically representative tissue areas of each ‘donor’ tissue block and brought into one recipient paraffin block (3×2.5 cm) using a semiautomated tissue arrayer (Galileo TMA, Milan, Italy).

### Histological analysis and immunohistochemistry

For light microscopy, tissues were fixed by immersion in 10% formalin and embedded in paraffin by standard procedures; 4 μm sections were stained with haematoxylin and eosin (H&E) or processed for immunohistochemistry. The classical avidin–biotin peroxidase complex (ABC) procedure was used for immunohistochemistry. The sections were incubated overnight with antibodies against CCDC6 at 1: 200 dilution. The following controls were performed: (a) omission of the primary antibody; (b) substitution of the primary antiserum with non-immune serum diluted 1: 500 in blocking buffer; (c) addition of the target peptide used to produce the antibody (10^−6^ M); no immunostaining was observed after any of the control procedures. The antibody against the CCDC6 proteins is from Sigma-Aldrich, Co. LLC. (HPA-019051).

### Protein extraction and western blot analysis

Total cell extracts (TCE) were prepared with lysis buffer (50 mM Tris–HCl pH 7.5, 150 mM NaCl, 1% Triton X-100, 0.5% Na Deoxycholate, 0.1% SDS) and a mix of protease inhibitors. Protein concentration was estimated by a modified Bradford assay (Bio-Rad). Total proteins were prepared as described [22]. Membranes were blocked with 5% TBS-BSA proteins and incubated with the primary antibodies. Immunoblotting experiments were carried out according to standard procedures and visualized using the ECL chemiluminescence system (Amersham/Pharmacia Biotech). As a control for equal loading of protein lysates, the blotted proteins were probed with antibody against anti-γ-tubulin protein.

### Real time PCR

Total RNA was isolated using TRI-reagent solution (Sigma) according to the manufacturer’s instructions and treated with DNase I (GenHunter Corporation, Nashville, TN, U.S.A.). RNA (1 μg) was reverse-transcribed using a mixture of poly-dT and random exonucleotides as primers and MuLV RT (PerkinElmer, Boston, MA, U.S.A.). PCR reverse transcription was performed according to standard procedures (Qiagen). qRT-PCR analysis was performed using the follows primers annealing at CCDC6 amino-terminus: Fw: ggagaaagaaacccttgctg and Rv: tcttcatcagtttgttgacctga. To calculate the relative expression levels we used the 2−ΔΔCT method. Primers for Beta-actin were used for normalization of qRT-PCR data [23].

### Fluorometric determination of Reactive Oxygen Species (ROS)

The production of ROS was measured using the 5,6-carboxy-2′-7′-dichlorofluorescein-diacetate, DCFH-DA, fluorometric method, which is based on the ROS-dependent oxidation of DCFH-DA to DCF (Molecular Probes, The Netherlans). Control and transfected GC1 cells, after H_2_O_2_ exposure where indicated, were treated with DCFH-DA (20 μM) for 30 min at 37°C in the dark. Intracellular ROS production was measured with a spectrofluorometer (SFM 25; Kontron Instruments, Japan). A positive control was obtained by incubating GC1 cells with H_2_O_2_ at 10 μM for 1 hour.

## Results

### CCDC6 expression in mouse testicular cells

In order to define the cells in which CCDC6 is expressed in the normal testis, immunohistochemical analysis for this protein was performed on serial sections of the mouse testis. The CCDC6 protein was widely expressed in the germinal epithelium, mostly in the spermatogonial cells found at the basal compartment of the seminiferous epithelium, where they adhere to the basement membrane, while less so in the spermatocytes and spermatids. The Sertoli cells, essential components of the niche where they physically support the spermatogonial cells and provide them with growth factors, also expressed a good amount of the CCDC6 gene product, while it was not detectable in the spermatozoa (Figure 1A). Importantly, we checked that the antiserum used in this study fulfilled the criteria of specificity. In particular, immunoadsorption tests revealed that the labeling was totally blocked by preincubation of the antibody with 10^-6^ M of the cognate peptide (data not shown).

**Figure 1:** **CCDC6 expression in adult mouse testis. (A)** Immunohistochemical staining for CCDC6 protein in adult mouse testis (LSAB tecnique). A representative seminiferous tubule showing staining in the basal germ cells (arrow heads), Sertoli cells and Leydig cells. **(B)** Distribution of CCDC6 protein in mouse testicular cells. Western blot analysis of CCDC6 protein in mouse adult testis (lane 1), interstitium (lane 2), Sertoli cells (lane 3) and normal mouse germ cells (lanes 4–7) (40 μg/lane). Whole lysates were detected by western blotting with anti-CCDC6 polyclonal serum or with anti-ERK1 antibodies used as an internal standard. ERK1 antibodies recognize both ERK1 and ERK2, which are expressed at similar levels in all cell types with the exception of spermatozoa. Anti-tubulin hybridization is shown as loading control.

Next, we confirmed the differential expression of CCDC6 in the different cell types in the mouse testis, by Western Blot analysis of cell extracts from the adult mouse testis fractionated in interstitial, Sertoli, spermatogonia, spermatocytes, spermatids and spermatozoa. Immunoblot analysis performed on cell types enriched in the different types of germ cells showed a single product migrating as a 65 kDa protein (Figure 1B). Among germ cells, CCDC6 was well expressed in the spermatogonia, less abundant in the spermatocytes and spermatids and absent in the spermatozoa (Figure 1B), in agreement with the immunohistochemical results. Moreover, the CCDC6 protein was present in the interstitial, at low levels, and the Sertoli extract cells (Figure 1B).

### CCDC6 silencing in the GC-1 spermatogonia increases the resistance to peroxide-induced apoptosis

We have previously reported that CCDC6 overexpression is able to induce apoptosis [9]. Conversely, we have shown that several CCDC6 mutants or CCDC6 depletion protected cell viability from multiple and diverse apoptotic stimuli [9,10]. Recently, it has been reported that primary testicular germ cells are prone to apoptosis at very low concentrations of H_2_O_2 _[24]. Next, we investigated CCDC6 expression in the GC1 cells, derived from immortalized type B murine germ cells that were found to express good levels of CCDC6 (Figure 2A, right). In order to investigate if the loss of CCDC6 could affect hydrogen peroxide-induced apoptosis in CCDC6-expressing primordial GC1 cells, we silenced its expression by the transient transfection of specific shRNAs directed against murine CCDC6 and exposed the cells to different doses of hydrogen peroxide for 1 hour (Figure 2A, right). We observed a reversion of an antiproliferative effects following hydrogen peroxide exposure in CCDC6 silenced- compared to control GC1 cells. (Figure 2A, left). Pro-apoptotic stimuli, like reactive oxygen species (ROS), are able to activate the intrinsic pathway of apoptosis by inducing mitochondrial membrane permeabilization and the release of cytochrome c in the cytosol [25]. Indeed, by western blot analysis, we observed that the oxidized form of cytochrome c was significantly decreased in GC1-shCCDC6, compared to controls (Figure 2A, right). Furthermore, we performed the Cytochrome C Releasing Apoptosis Assay that we show in Figure 2B. By this assay we found that 48 hours after the transient silencing of shCCDC6 and shCTRL in GC1 cells the cytochrome c release in the cytosol of the GC1 shCCDC6 cells showed a slightly increase, compared to the significant high levels detected in the shCTRL GC1 cells, following one hour exposure to 10 μM H2O2, after washing out the hydrogen peroxide and leaving the cells an additional hour before the lysis. The same filters were reprobed with a monoclonal antibody against cytochrome oxidase subunit IV (COX IV) which is a mitochondrial marker, and then with the anti-tubulin antibody, which is a cytosolic marker. The absence of COX IV in the cytosolic samples confirmed the absence of mitochondrial contamination in the cytosolic fractions (Figure 2B, left). Finally we sorted out the relative intensity of the cytochrome c in the cytosolic and mitochondrial fractions normalized against the tubulin and the COX IV markers, respectively, in shctrl and in sh CCDC6 GC1 cells, by densitometric analyses of three independent experiments (Figure 2B, right).

**Figure 2:** **Peroxide sensitivity in CCDC6 silenced GC1 cells. (A)** Left side: percentage of cell viability evaluated by MTT analysis on GC1 shCCDC6 or sh ctrl cells not treated or treated for 1 hour with H2O2. Right side: CCDC6 and Cytochrome C immunoblots of GC1 shCCDC or sh ctrl cells, not treated or treated with H2O2. **(B)** Protein extracts from cytosol (C) and mitochondria (M) of shctrl and shCCDC6 cells untreated or treated with H2O2 as indicated were assayed for Cytochrome c by western blot analysis. Tubulin was used as cytosolic marker and COX IV as a mitochondrial marker. Densitometric acquisition are shown from three separate experiments. *p > 0,05 vs untreated shCTRL and shCCDC6 cells **(C)** WB analysis from GC1 shCCDC6 or sh ctrl lysates from cells not treated or treated with H2O2. The blots are representative of three independent experiments. **(D)** Caspase 3 activity was evaluated in GC1 cells, shCCDC6 or sh ctrl, not treated or treated with H2O2. The plotted values represent the mean +/- s.e.m. of three independent experiments. **(E)** Whole cell lysates from GC1 shCCDC6 or sh ctrl cells, and from GC1 cells overexpressing CCDC6T434A or the empty vector, treated with H2O2 (10 μM) or untreated were immunoblotted with anti-CCDC6 or anti-myc. Anti- γH2AX and total H2AX are shown. **(F)** GC1 cells, depleted or not depleted for CCDC6, were exposed to 50 μM H2O2 for 30 minutes and ROS intracellular levels were evaluated by the DCFH-DA fluorometric method. **(G)** GC1 cells overexpressing CCDC6T434A or the empty vector were exposed to 50 μM H2O2 for 30 minutes and ROS intracellular levels were evaluated by the DCFH-DA fluorometric method. In **F** and **G** data are representative of three separate experiments. # p > 0.05 vs control. Immunoblot of anti-tubulin is shown in **A**, **C** and **E**.

To determine whether the H_2_O_2_-induced redox imbalance and the subsequent GC1 cell apoptosis were associated with changes in pro- and anti-apoptotic proteins, the expression of these proteins was analyzed by western blot. Bad protein showed lower levels in the GC1-shCCDC6 transfected cells compared to the sh-control transfected cells, after 1 hour treatment with 10 μM H_2_O_2_. The anti-apoptotic Bcl2 protein levels were found to be increased after 10 μM hydrogen peroxide treatment in the CCDC6-depleted GC1 cells, compared to the CCDC6-proficient cells. In addition, we observed that the levels of Caspase 3 and of the cleaved PARP-1 proteins were reduced in the CCDC6-silenced cells compared to the controls. In these experiments, the effects were more evident at 10 μM than at 1, 2 and 5 μM doses of H_2_O_2_, according to the efficiency of the transient silencing (Figure 2C; Additional file 2: Figure S2). To investigate whether CCDC6 silencing was able to confer protection by H_2_O_2_ induced apoptosis in testicular germ cells, we studied caspase −3 activity. We found that caspase −3 activity was reduced in shCCDC6 compared to shCTRL GC1 cells, upon 10 μM H_2_O_2_ treatment for 1 hour (Figure 2D).

### CCDC6 silencing in the GC-1 germ cells decreases reactive oxygen species production

We reported that stable CCDC6 depletion in HeLa cells affected the phosphorylation of histone H2AX on S139, upon IR and etoposide exposure [11]. In the same cells, CCDC6 silencing affects the levels of histone H2AX phosphorylation, upon H_2_O_2_ treatment (data not shown). Interestingly, in the stable CCDC6-interfered HeLa cells, the re-expression of the wild type protein but not of the CCDC6 protein mutated in the T434A residue, an ATM kinase phosphorylation target, restored pS139_H2AX levels in response to genotoxic stress [11]. Indeed, also in the GC1 cells, the transient silencing of CCDC6 impaired pS139_H2AX detection upon low doses of H2O2 treatment, compared to control cells (Figure 2E). Notably, the overexpression of the CCDC6 T434A mutant, that behaved as a dominant negative of the wild type protein, affected the phosphorylation status of the histone H2AX in the absence or presence of H_2_O_2_, in comparison to the empty vector transfected cells (Figure 2E). These observations therefore suggested that the recognition site for the ATM kinase in CCDC6 was also important in response to DNA damage induced by oxidative stress. By immunoblot analysis of CCDC6, we could also observe that the protein was stabilized in response to H_2_O_2_ in the sh-ctrl and in the empty vector transfected GC-1 cells, compared to the T434A overexpressing cells, where the H_2_O_2_ treatments did not stabilize the CCDC6 protein (Figure 2E). As a control, in the lanes where CCDC6 was silenced in the GC1 cells (−/+H_2_O_2_), the anti-CCDC6 hybridization allows a verification of the efficiency of the silencing (Figure 2E). Overall, these experiments have showed that, in the GC1 cells, the loss of CCDC6 or its functional impairment by mutation of a single residue limited the amount of S139_pH2AX that then influenced the sensing of DNA damage induced by H_2_O_2_, relative to the control cells.

Finally, to evaluate whether an altered redox state could be responsible for the pro-survival effects observed when CCDC6 is depleted, we measured the intracellular levels of ROS, in response to H_2_O_2_ exposure. In the GC1 cells the transient silencing of CCDC6 produced lower levels of ROS, compared to control (*p ≤ 0.05) (Figure 2F), as judged by the fluorescence signal detection following the interaction between the DCFH-DA probe and ROS. In the same cells, the transient expression of the mutant CCDC6 T434A counteracted the ROS production, compared to the control (# p ≤ 0.05) (Figure 2G).

### CCDC6 and DDR protein expression in testicular seminomas

In order to assess the CCDC6 expression in human testes and testicular germ cell tumors, in the first instance we tested twenty testicular seminomas, including IGCNU, one yolk salk tumor and five embrionary carcinomas and the corresponding normal tissues for CCDC6 expression by immunohistochemistry with an anti-CCDC6 specific monoclonal antibody. The representative immunohistochemical stainings are shown in Figure 3. CCDC6 was virtually undetectable (<2.0% of cells) in the nuclei of the neoplastic cells in the seminomas. In the testicular tissues adjacent to the tumour, normal or atrophic and not affected by neoplastic transformation, it was possible to appreciate the CCDC6 positivity mainly in the nucleus of the spermatogonial cells identified, on the basis of the morphological features, at the basal layer of the tubules. The CCDC6 staining decreased proceeding from the basal layer to the lumen (Figure 3). The Sertoli and Leydig cells showed both cytosolic and nuclear staining. IGCNU was appreciable in nearly all tumour samples (90%). In all these cases, the neoplastic cells present in the IGCNU showed weak (<3%) CCDC6 nuclear stainings similar to normal spermatogonial cells (Figure 3, middle). In the yolk salk tumor and in the embrionary carcinomas the immunostaining for CCDC6 was nearly undetectable (Figure 3, bottom).

**Figure 3:** **Immunohistochemical staining for CCDC6 in human testis.** Immunohistochemical staining for CCDC6 in normal testis, normal testis adjacent to an area of seminoma, IGCNU (intratubular germ cell neoplasia unclassified), seminoma (top to bottom), yolk sac tumor and embyonary carcinoma. Immunoreactivity for CCDC6 is mainly detected in nuclei of primordial germinal cells and Sertoli cells of normal testis; nuclear CCDC6 reactivity is almost absent in IGCNU, in seminoma, in yolk sac tumour and in embryonal carcinoma. Magnifications are respectively: 200×, 106×, 250×, 250×, 250×, 250×.

In order to evaluate the activation of the DDR machinery in the same set of samples, we investigated the immunostaining for pS1981_ATM, the activated form of a key upstream regulator that controls most DDR events; the staining for pT68_Chk2, a central mediator of DDR that resulted barely detectable in IGCNU and in primary tumours was also analysed (Figure 4). Histone H2AX phosphorylation, a downstream chromatin modification linked to the generation of double-strand breaks (DSBs), showed a certain grade of positivity in normal germ cells (Figure 4). Such positivity for histone phosphorylation, visible also in some of the testicular seminomas analysed, was likely to be due to replicative stress in the spermatocyte population in the different phases of differentiation present in the tumour and healthy tissues, as already reported [8]. At the end, we checked the expression of MDC1, recently emerged as an important spatio-temporal regulator of the genome integrity maintenance close to the top of the DNA machinery signaling and lesion proceeding cascades [25,26]. An aberrant reduction or a lack of MDC1 has been reported in a significant proportion of carcinomas supporting its candidacy as a tumor suppressor [26]. In contrast to carcinomas, almost no activation or loss has been found in testicular germ cell tumours [27]. We also found no substantial variation in the expression of MDC1 among our cases: a definite nuclear staining for MDC1 was in fact present in the normal seminiferous tubules (Figure 4), as reported [28], in the IGCNU (middle part of Figure 4) and in the invasive seminomas. Next, we confirmed all the observations we obtained by IHC staining also by Western blot analysis of 10 primary tissues obtained from a different set of patients. As shown in the representative samples of Figure 5, CCDC6 was expressed at very low levels in almost all seminomas and was virtually absent in teratocarcinomas and in embryonal carcinomas, compared to the normal samples (Figure 5). Moreover, we investigated the CCDC6 protein expression in the TCam-2 cell line, derived from a human seminoma. By immunoblot analysis, protein hybridization showed a low expression of CCDC6 in the TCam2 seminoma cells, similar to the primary tumours (Figure 5A). Quantitative real time PCR analysis showed low levels of transcripts for CCDC6 in these cells, compared to the expression levels detected in the GC1 cells (Figure 5B), suggesting that the loss of CCDC6 in the neoplastic seminoma cells might not be dependent on a post-transcriptional mechanism. Next, in order to investigate the level of activation of the DDR molecules in the seminoma TCam2 cells, we performed Western Blot hybridization with specific antibodies against pS1981_ATM (pATM), pT68_Chk2 (pChk2) and pS139_H2AX (γH2AX) observing a barely detectable signal, after 1 hour treatment with 10 μM H2O2 for all these DDR activation markers in TCam2 cells, compared to the levels observed in the GC1 normal testicular germ cells [18] (Figure 5C).

**Figure 4:** **Immunohistochemical staining for the DDR molecules in seminoma, IGCNU and normal testis.** pS1981-ATM, pT68-CHK2, γH2AX and MDC1 show weak to absent, focal nuclear positivity. Immunostaining for ATM, CHK2 and H2AX shows a strong nuclear reactivity in all the samples. Magnifications are 250× for pS1981ATM and ATM in seminoma, 200× for CHK2 and γH2AX in normal trestis, 150× for the remaining.

**Figure 5:** **Analysis of CCDC6 expression in normal human testis and testicular germ cells tumors. (A)** 40 ug of total tissue lysates were resolved on 10% SDS-PAGE transferred onto nitrocellulose filters and western blotted with α-CCDC6 antibody. NT, normal testis; lanes 2–6: seminomas; lane 7, teratoma; lane 8, embryonal carcinoma; lane 9, TCAM2 seminoma cell line. Anti-actin hybridization is shown as loading control. The blots are representative of three independent experiments. **(B)** Top: CCDC6 relative expression in TCAM2 and GC1 cells analysed by qRT-PCR. Data are the mean +/− SD of three independent experiments. Bottom: CCDC6 expression in the unique TCAM2 seminoma cells and GC1 Cells. Whole lysates were detected by western blotting with anti-CCDC6 antibody. **(C)** the activation of the molecules of the DNA Damage Response were monitored using the anti-pS1981_ATM (pATM), the anti-pT68_Chk2 (pChk2), and the anti-pS139_H2AX (γH2AX). Total ATM, Chk2 and H2AX are shown. Before lysis, the cells have been treated 1 hour with H_2_O_2_ (10 μM), and after washing out the hydrogen peroxide the cells have been left an additional hour before the lysis. Anti-tubulin hybridization is shown as loading control.

### TMA based analysis of CCDC6 expression in testicular tumors

To confirm our findings and in order to extend the CCDC6 expression analysis in a larger set of human testicular samples, we took advantage of the tissue microarray (TMA) technique. TMA is a reliable and representative technology that allows the in situ analysis of tumoural and normal tissue samples in a high-throughput and internally controlled format. We screened a total of 87 human testicular tumours of different histotypes and 10 paired normal tissues using TMA. In Table 1, the TMA composition of the tumours derived from the testicular germ cells is listed. The CCDC6 protein expression was reduced in the tumours as witnessed by the low signal obtained per single cells and by the decreased number of cells/field stained with the anti-CCDC6 antibody.

**Table 1:** Germ cell tumors TMA composition

**Tumoral hystotypes**	**Total number (87)**	**Percentage %**	**CCDC6**	**γH2AX**
Seminoma	46	53	39/46 -	+/-
			7/46 +/-	-
Embryonal carcinoma	15	17,1	15/15 -	+/-
Mixed carcinoma	20	23	20/20 +/-	+/-
Teratoma	5	5,8	2/5 +/-	+/-
			3/5 -	-
Yolk sac tumor	1	1,1	1 /1 -	+/-

In all the testicular seminomas and embryonal carcinomas, we observed a low to absent nuclear positivity for CCDC6 (Figure 4). Together with the CCDC6 protein, we also assessed the engagement of the DDR machinery in the same tumours and in their normal counterparts, when available. Specifically, we investigated the DDR-signaling cascade at three nodal points: pS1981_ATM, the activated form of a key upstream regulator that controls most DDR events; pT68_Chk2, a central mediator of DDR and pS139_H2AX, the chromatin event following DSBs. By these markers we observed that DDR machinery activation resulted virtually absent in the human testicular tumours analyzed: little evidences of the activated checkpoint kinases ATM or Chk2 was indeed observed (data not shown), in contrast to some cells that showed activated pS139_H2AX (Table 1).

## Discussion

The incidence of testicular germ-cell cancer, the most common malignancy in young men, has recently shown an alarming rise in the industrialized countries. This trend, together with the worrying decline in male reproductive health, and the fascinating biology of the germ cells and germ-cell tumours (GCTs), have stimulated an increasing number of studies to better understand the cellular and molecular biology of reproductions, and the molecular pathogenesis of testicular cancer [29-32].

The genome locus for CCDC6 is commonly rearranged in various tumours and, despite the emerging role for CCDC6 as a tumour suppressor, possibly controlling intra S-phase [33] and G2/M cell cycle checkpoints and DNA repair [11], its biology and pathology remain largely unexplored. A few CCDC6 somatic mutations have been reported in some tumours (http://www.sanger.ac.uk/genetics/CGP/cosmic), but they are still in need of characterization. Also, there are no data on the abundance, localization or cell-type specificity of the CCDC6 protein in human tissues and tumours. The reasons which led us to choose spermatogenesis and testicular cancer to study CCDC6 include: (i) that CCDC6 is predicted as downregulated in germ cell tumours (by the analysis of the ArrayExpress Archive database), (ii) the occurrence, in the same tissue, of both mitotic and meiotic cell cycles, (iii) the high frequency of programmed DSBs as an essential part of genetic recombination during meiosis and (iv) the oxidative DNA damage envisaged as emerging mechanism of carcinogenesis in this tissue [5,34].

For the purpose of assessing CCDC6 expression in a large series of human testicular tumour samples, we analysed 20 primary tumours by also taking advantage of the TMA technique, that provides a great opportunity to easily analyze, store and share IHC data of a large number of samples [35-37]. Primary tumours and TMA immunostaining investigations of CCDC6 expression demonstrated that CCDC6 is severely downregulated in all the different testicular tumours analyzed. Moreover, the analysis of IGCNU, the presumed precursor lesion of germ cell tumours, showed a barely detectable nuclear staining for CCDC6, suggesting that CCDC6 loss might represent an early event during cancer development in the testis. Still, the observation that there is no significant difference in CCDC6 at mRNA and protein levels in the unique seminoma TCAM2 cell line reinforces the hypothesis that the loss of CCDC6 expression might occur as a transcriptional event. Since no fusions or mutations involving CCDC6 have been reported in testicular cancer, so far, we cannot rule out the existence of other mechanisms, such as promoter methylation that could contribute to inactivate CCDC6 in TGCTs. Nevertheless, we can assume that in different tissues, other than the testis, CCDC6 may be inactivated or lost by different mechanisms, such as post-translational modifications, and also at different stages of tumour development, initiation or progression. Further investigations are in progress in different tumour histotypes in order to clarify these critical points.

By analyzing the murine testicular cell population by IHC and by cell population fractionation, we observed a specific expression of CCDC6 in the spermatogonial cells. In contrast, CCDC6 was weakly expressed or undetectable in the spermatocytes at different stages of meiosis, and virtually negative in the post-meiotic stages of spermatogenesis. The progressively decreasing levels of CCDC6 during the spermatocytic differentiation process could reflect the different levels of control needed for the mitotically proliferating testicular cells rather than during meiotic recombination where CCDC6 could probably induce inadequate apoptosis and undermine spermatogenesis.

DNA damage response is emerging as a physiological anti-cancer barrier in early stages of cancer development in several types of solid cancer, derived from somatic cells, as opposed to the exceptional paucity of such constitutive activation in human testicular germ cell tumours (TGCTs) [8]. Indeed, we detected low levels of CCDC6 and confirmed a very low activation of DDR-controlling molecules in the testicular germ cells tumours that we analyzed.

Interestingly, complex anti-oxidant defense systems have been reported in rat and human testes [34,38], while oxidative DNA damage is emerging as a mechanism of carcinogenesis [5,39]. Several studies have, in fact, also documented the presence of high levels of oxidative damage in A-T patients [40]. Recently, the ATM kinase has been reported to promote anti-oxidant defense and DNA repair, and, consequently, has been involved in response to oxidative stress [41].

It has been reported that, in primary testicular germ cells, the treatment with low doses of H_2_O_2_ is associated with a rise in oxidative stress and an induction of apoptosis [24]. H_2_O_2_ is a by-product of the cell metabolism and its cellular levels and maintenance are constantly under homeostatic regulation. As the major pathway of cell removal from the testis is through apoptosis, it is reasonable to assume that the redox status may either trigger or block the apoptotic death program depending on the severity of the oxidative stress. In this study, we first demonstrated that treatment of the GC1 cells with low doses of H_2_O_2_ induced apoptosis. Moreover, we found that, upon H_2_O_2_ treatment, the silencing of CCDC6 or the mutation in the recognition site for the ATM kinase in primary GC1 germ cells increases the rate of survival, impairs the phosphorylation of histone H2AX on S139, affects ROS production and makes the cells more resistant to oxidative damage. Since we have previously reported that CCDC6 could be considered a stress response protein participating to the control of genome stability [11], we can hypothesize that CCDC6 loss or impairment could also represent a mechanism to protect the cells from oxidative stress [9].

## Conclusions

In conclusion, our results suggest that the loss of CCDC6 in tumour testes could represent a specific event that helps testicular germ cell tumours formation. Moreover, defects in the DDR machinery could account for the beneficial effects of radio and/or chemo-therapy in association with surgical treatment in these tumours. However, we believe that a recurrence of the disease, even at low frequency, could be generated by a sub-population of tumor germ cells still able to activate the DDR. Therefore, we hypothesize that CCDC6 usage as a marker of cell population resistance could eventually favour a personalized treatment choice.

## Competing interests

The authors declare that they have no competing interests.

## Authors’ contributions

SS and AC designed the experiments. VL, CL, FM, FE and FM performed most of the experiments. SS, GI and MS performed the immunostainings and discussed the results. RF, PC and AF provided reagents and insightful comments on this work. AC analysed the experiments and wrote the manuscript. All authors reviewed and edited the manuscript drafts and agreed to the final version of the manuscript.

## Pre-publication history

The pre-publication history for this paper can be accessed here:

http://www.biomedcentral.com/1471-2407/13/433/prepub

## Supplementary Material

Additional file 1: Figure S1 GC-1 cells were transfected with mission shCCDC6 or a control non-targeting scrambled sh, after 48h were treated with H_2_O_2_ at different doses (range of 1, 2, 5, 10 and 50 μM) for 30 min and 1h, as indicated. After washing out the hydrogen peroxide we have left the cells an additional hour before processing them. 20 ml of Promega’s CellTiter 96 AQueous One Solution (Promega) were then dispensed into each well and absorbance at 595nm was measured to evaluate cell viability. Data reported are the average +/− s.d. of three independent experiments performed in sextuplicate. Click here for file

Additional file 2: Figure S2 Densitometric analysis has been performed by Image J software; the results of three independent experiments were plotted as percent of the ratio between the CCDC6 and tubulin intensity, respectively, as indicated. Error bars, +/− SD. P values are shown. Click here for file
